# Cheap and rapid in-house method for direct identification of positive blood cultures by MALDI-TOF MS technology

**DOI:** 10.1186/s12879-019-3709-9

**Published:** 2019-01-18

**Authors:** Maya Azrad, Yoram Keness, Orna Nitzan, Nina Pastukh, Linda Tkhawkho, Victoria Freidus, Avi Peretz

**Affiliations:** 1 Clinical Microbiology Laboratory, Baruch Padeh Medical Center, Poriya, Israel; 2 Clinical Microbiology Laboratory, Ziv Medical Center, Zefat, Israel; 3 Clinical Microbiology Laboratory, Emek Medical Center, Afula, Israel; 4 Faculty of Medicine, Bar Ilan University, Galilee, Israel; 5 Unit of Infectious Diseases, Baruch Padeh Medical Center, Poriya, Israel

**Keywords:** MALDI-TOF MS, Blood culture, SepsiTyper kit, BACTEC™ FX system, Bacteria

## Abstract

**Background:**

Rapid and accurate pathogen identification in blood cultures is very important for septic patients and has major consequences on morbidity and mortality rates. In recent years, matrix-assisted laser desorption ionization–time of flight mass spectrometry (MALDI-TOF MS)-based technology has become useful for highly specific and sensitive identification of bacteria and yeasts from clinical samples including sterile body fluids. Additional in-house methods enabled direct identification from blood cultures following various preparation protocols.

**Methods:**

Blood culture (5 ml) was harvested from each positive bottle following growth identification by BACTEC™ FX system and transferred into a VACUETTE® Z Serum Sep Clot Activator tube containing an inert gel, which following centrifugation separates microorganisms from the blood cells. We used MALDI-TOF MS analysis for identification of microorganisms collected from the gel surface.

**Results:**

Positive blood culture bottles (186) were collected. In comparison with the routine method, 99% (184/186) and 90% (168/186) of the isolates were correctly identified by the SepsiTyper kit and the in-house method, respectively. We found high concordance (Pearson coefficient = 0.7, *p* <  0.0001) between our in-house method and the SepsiTyper kit. Additionally, high correlation was found in sub-groups of identified bacteria, with Pearson coefficients of 0.77 (*p* <  0.0001), 0.67 (*p* <  0.0001), and 0.73 (*p* <  0.007) for Gram negative, Gram positive, and anaerobic bacteria, respectively.

**Conclusions:**

Our in-house method was found to be in good agreement with the SepsiTyper kit. Considering the low costs and the rapid and easy implementation of this procedure, we propose our in-house method for the direct identification of bacteria from blood cultures.

## Background

Presence of microorganisms in the bloodstream is a life-threatening situation that requires rapid identification and treatment. Pathogen identification is of great significance, enabling adjustment of antibiotic care.

In most clinical microbiology laboratories, the traditional method for microbial identification includes sampling of a blood specimen from the positive blood culture, subculturing it onto solid agars for 18–24 h, and bacterial identification according to biochemical features and antimicrobial susceptibility testing. The primary disadvantage of this method is that causative pathogen identification is performed only after colony growth and isolation, which leads to a prolonged turnaround time, especially when handling slow growing microorganisms such as anaerobic bacteria and yeasts. As time from diagnosis to appropriate antimicrobial care strongly influences mortality, shortening the turnaround time of pathogen recognition is extremely important [1, 2].

In recent years, matrix-assisted laser desorption ionization–time of flight mass spectrometry (MALDI-TOF MS)-based technology has become useful for highly specific and sensitive identification of bacteria and yeasts from clinical samples. In this technique, a laser beam irradiates microorganism colonies and ionizes their proteins. As each microorganism has a different ionized protein profile, a different mass spectrum is created by the MALDI-TOF MS device. Whenever a new sample is subject to MS analysis, the software compares its profile to a database in order to define the microorganism. The first devices enabled pathogen recognition from one colony, grown on solid agar [3]. Later, new protocols were developed for identification of microorganisms directly from sterile body fluids such as cerebrospinal fluid, in order to save the culturing time [4]. Additional in-house methods enabled direct identification from blood cultures following various preparation protocols. Most of these protocols require hemolysis of red blood cells [2] and several blood centrifugations for the separation of blood cells and microorganisms [1, 2]. Along with laboratory-developed procedures, several commercial kits were developed, saving the handling time of solution preparation and additional equipment purchase. One such kit is the MALDI SepsiTyper Kit (Bruker Daltonics, Bremen, Germany), which was described in various studies as an efficient and successful tool for identification of bacteria and yeasts directly from blood cultures [5]. Successful microbial identification in this assay, as well as in others, depends on the bacterial amount that is collected from the culture pellet. The primary disadvantage of ready-to-use kits is their high cost.

In the current study we compared bacteria and yeast identification by MALDI SepsiTyper with a simple and cost-saving method using a VACUETTE® Z Serum Sep Clot Activator tube, which is frequently used in clinical laboratories and enables separation of microorganisms from blood cells.

## Methods

### Positive blood culture collection

The research was performed at the Baruch Padeh Medical Center, Poriya, in northern Israel. During January to April 2016, we collected positive blood cultures (BCs) from patients who were admitted to the hospital; these were sent to the clinical microbiology laboratory. Each BC bottle that arrives to the clinical microbiology laboratory is incubated in the BACTEC™ FX system **(**BD Diagnostics, Sparks, MD) for microorganism growth monitoring.

Following microorganism growth identification by the BACTEC™ FX system, the blood culture media was collected from each bottle and subjected to Gram staining. For this study, a total of 186 positive BCs were collected from 93 patients. These 186 BCs were selected only based on Gram staining in order to confirm the presence of one organism per BC bottle; 104 of these BCs were collected in Plus Anaerobic/F Culture Vials (BD Diagnostics, Sparks, MD) and 82 were collected in Aerobic/F Culture Vials (BD Diagnostics, Sparks, MD).

### Identification by the routine method

Following microorganism growth identification by the BACTEC™ FX system and Gram staining, the blood culture media was subcultured onto solid growth media including blood, MacConkey, and chocolate agar (BD Diagnostics, Sparks, MD) (drop culture). Agar plates were incubated at 36 ± 1 °C in 5% CO_2_ for 18–24 h. In accordance with clinical data of the patient and/or Gram staining, in case of suspected anaerobic bacteria, the sample was additionally subcultured on CDC and blood-amikacin agars (Hy-Laboratories Ltd., Israel), which were incubated at 37 °C for 5 days, under anaerobic conditions. Whenever Gram stain indicated presence of yeasts, the sample was additionally subcultured on CHROMagar Candida (Hy-Laboratories Ltd., Israel), which was incubated at 37 °C for 48 h. Following incubation, isolated colonies were spotted onto a MALDI-TOF MS target plate (Bruker Daltonics, Bremen, Germany) and subjected to MALDI-TOF MS analysis, as described below.

### Identification by MALDI SepsiTyper kit

The MALDI SepsiTyper kit was used simultaneously with the routine method, following the Gram staining. BC media (1 ml) was harvested from each positive BC and transferred into an Eppendorf tube; 200 μl of lysis buffer was added and mixed for 10 s. Following centrifugation (2 min, 13,000 rpm), supernatant was discarded and pellet resuspended in 1 ml of washing buffer. After a second centrifugation (1 min, 13,000 rpm), supernatant was discarded and pellet was resuspended in 300 μl of HPLC-grade water. After addition of 900 μl ethanol, the tube was centrifuged (2 min, 13,000 rpm). Supernatant was discarded and the pellet was subjected to additional centrifugation (2 min, 13,000 rpm). Supernatant was discarded and the pellet was air-dried for 5 min at room temperature. Then the pellet was resuspended in 2–50 μl of 70% formic acid (Merck, Herzliya, Israel) and equal quantity of acetonitrile (Merck, Herzliya, Israel). Following centrifugation (2 min, 13,000 rpm), 1 μl of the supernatant was deposited onto MALDI target plate (Bruker Daltonics, Bremen, Germany) for MALDI-TOF MS analysis, as described below.

### Identification by in-house method

The in-house method was used simultaneously with the routine method, following the Gram staining. BC media (5 ml) was harvested from each positive BC and transferred into VACUETTE® Z Serum Sep Clot Activator tube (Greiner Bio-One**,** North Carolina, USA). This tube contains an inert gel, which, after centrifugation, physically separates the serum and the blood cells. Each tube was centrifuged (10 min, 3000 rpm) and supernatant carefully discarded. Pellet was taken from the surface of the separating gel and resuspended in 1 ml saline. Following centrifugation (2 min, 13,000 rpm), 1 μl of the supernatant was deposited onto MALDI target plate (Bruker Daltonics, Bremen, Germany) for MALDI-TOF MS analysis, as described below.

### MALDI-TOF MS analysis

Following drying of spotted colonies (routine method) or bacterial pellet (in-house method and SepsiTyper kit) on a MALDI-TOF MS target plate (Bruker Daltonics, Bremen, Germany), 1 μl of alpha-cyano-4- hydroxycinnamic acid (HCCA) matrix solution was placed onto each spot and air-dried. MALDI-TOF MS analysis was performed by Microflex LT system (Bruker Daltonics, Bremen, Germany) with MALDI BIOTYPER 3.3 (Bruker Daltonics) software.

Analysis results are presented as a score. According to manufacturer’s instructions, score < 1.7 indicates no reliable identification, a score between 1.7 and 1.999 indicates identification to the genus level, and a score ≥ 2 indicates identification to the species level.

The methods that were used in the study are summarized in Fig. 1.

**Fig. 1:** Flow diagram of the three methods that were used for the identification of positive blood cultures (routine method, in-house method, and SepsiTyper kit)

### Statistical analysis

Pearson correlations coefficients were calculated for testing the agreement between the SepsiTyper kit and the in-house method in quantitative (continuous) scores by group and overall.

Correct identification rates were calculated as follows: The identification results of each method (the SepsiTyper kit and in-house method) were compared to the identification results of the routine method (from isolated colonies).

The correct identification rates are the number of isolates that were correctly identified by either the SepsiTyper kit or the in-house method (regardless of the identification score), divided by the overall number of isolates (in sub-groups and overall).

Statistical significance was determined with *p* value < 0.05. The data was analyzed using the SAS® version 9.3 (SAS Institute, Cary, NC).

## Results

During the study period, 186 positive BCs were collected from 93 patients. All 186 BCs were identified by the routine laboratory method. Overall, 88 (47.3%) Gram positive, 79 (42.5%) Gram negative, 7 (3.8%) yeasts, and 12 (6.4%) anaerobic bacteria were identified. Table 1 presents microorganism identification results of the positive BCs that were analyzed by MS following SepsiTyper kit and in-house method, and the analysis scores.

**Table 1:** Results of MS analysis for microorganisms’ identification in positive blood cultures using SepsiTyper kit and in-house method

Species (as identified by the routine method)	N	SepsiTyper kit				In-house method			
		S^a^ < 1.7	1.7 ≤ S ≤ 1.999	S ≥ 2.0	No identification	S < 1.7	1.7 ≤ S ≤ 1.999	S ≥ 2.0	No identification
*Acinetobacter baumannii*	6	1	4	1		3	3		
*Bacteroides fragilis*	2	2	2			2			2
*Campylobacter fetus*	2	2				1			1
*Candida albicans*	5	1	3		1	3			2
*Candida tropicalis*	2	1	1						2
*Citrobacter freundii*	2		1	1		1		1	
*Citrobacter koseri*	4		2	2		2	2		
*Clostridium perfringens*	2		1	1		1	1		
*Corynebacterium amycolatum*	2		2			1			1
*Corynebacterium jeikeium*	1	1				1			
*Enterobacter aerogenes*	4		2	2		3	1		
*Enterobacter cloacae*	4		2	2		1	3		
*Enterococcus faecalis*	11	2	7	2		6	4		1
*Escherichia coli*	17		6	11		7	8	2	
*Fusobacterium nucleatum*	2	1	1			1			1
*Haemophilus influenzae*	3	2			1				3
*Klebsiella oxytoca*	2		2			2			
*Klebsiella pneumoniae*	11		6	5		3	8		
*Micrococcus luteus*	3		1	2		1	2		
*Morganella morganii*	2			2			2		
*Plesiomonas shigelloides*	3		2	1		2	1		
*Propionibacterium acnes*	4	1	3			3	1		
*Proteus mirabilis*	4			4			4		
*Providencia rettgeri*	4		2	2		1	2	1	
*Pseudomonas aeruginosa*	6		2	4		3	3		
*Serratia marcescens*	3			3		3			
*Staphylococcus aureus*	22		9	13		7	11	4	
*Staphylococcus capitis*	4		3	1		3	1		
*Staphylococcus epidermidis*	16	1	9	6		9	6		1
*Staphylococcus haemolyticus*	3	1	2			2			1
*Staphylococcus hominis*	4		1	3			4		
*Staphylococcus lugdunensis*	3		2	1		1	2		
*Stenotrophomonas maltophilia*	2		2			2			
*Streptococcus agalactiae*	2		1	1		1	1		
*Streptococcus dysgalactiae*	4	1	3			3			1
*Streptococcus gallolyticus*	2		2			2			
*Streptococcus pneumoniae*	5	1	2	2		2	2	1	
*Streptococcus pyogenes*	3	1	2			2			1
*Streptococcus sanguinis*	3		3			2			1

^a^ *S* Score

Out of 186 microorganisms, 88% (164/186) and 43.5% (81/186) were identified with a score ≥ 1.7 by SepsiTyper kit and by in-house method, respectively (Table 2); 50.5% (94/186) and 39% (72/186) of microorganisms were identified to the genus level (1.7 ≤ score ≤ 1.999) by SepsiTyper kit and by in-house method, respectively. Identification to the species level was obtained for 38% (70/186) and 5% (9/186) of microorganisms by SepsiTyper kit and by in-house method, respectively. No sample was misidentified by both methods.

**Table 2:** Results of MS analysis for microorganisms’ identification divided to microorganisms’ groups

Microorganism group	N	SepsiTyper kit				In-house method			
		S^a^ < 1.7	1.7 ≤ S ≤ 1.999	S ≥ 2.0	No identification	S < 1.7	1.7 ≤ S ≤ 1.999	S ≥ 2.0	No identification
Gram negative bacteria	79	5	33	40	1	34	37	4	4
Gram positive bacteria	88	9	50	29	0	43	33	5	7
Yeasts	7	2	4	0	1	3	0	0	4
Anaerobic bacteria	12	4	7	1	0	7	2	0	3
Total N (%)	186	20 (11)	94 (50)	70 (38)	2 (1)	87 (47)	72 (39)	9 (5)	18 (10)

### Gram positive bacteria

A total of 88 isolates were Gram positive bacteria. Out of 88, 90% (79/88) and 43% (38/88) of the isolates were identified with a score ≥ 1.7 by SepsiTyper kit and by in-house method, respectively (Table 2); 57% (50/88) and 38% (33/88) of the isolates were correctly identified to the genus level by SepsiTyper kit and by the in-house method, respectively; 33% (29/88) and 6% (5/88) of the isolates were identified to the species level by SepsiTyper kit and by the in-house method, respectively.

### Gram negative bacteria

Overall, 79 isolates were Gram negative bacteria. A score ≥ 1.7 was obtained for 92% (73/79) and 52% (41/79) of isolates, when analyzed by SepsiTyper kit and by the in-house method, respectively (Table 2).

Identification to the genus level was obtained for 42% (33/79) and 47% (37/79) of isolates when analyzed by SepsiTyper kit and by the in-house method, respectively. Identification to the species level was obtained for 51% (40/79) and 5% (4/79) of isolates, when analyzed by SepsiTyper kit and by the in-house method, respectively.

### Yeasts

Yeasts were isolated from 7 positive blood cultures. When analyzed by the in-house method, none of the isolates were identified with a score ≥ 1.7 (Table 2). When analyzed by the SepsiTyper kit, 4 out of 7 isolates were identified to the genus level. No identification to the species level was obtained with either of the methods.

### Anaerobic bacteria

A total of 12 anaerobic bacteria were isolated; 67% (8/12) and 16.6% (2/12) of isolates were identified with a score ≥ 1.7 by the SepsiTyper kit and by the in-house method, respectively (Table 2). Identification to the genus level was obtained for 58% (7/12) and 16.6% of the (2/12) isolates, when analyzed by the SepsiTyper kit and by the in-house method, respectively. One isolate (8%) was identified to the species level when analyzed by the SepsiTyper kit. No identification to the species level was obtained by the in-house method.

### Correct identification rates

Overall correct identification rates were 99% (184/186) and 90% (168/186) for SepsiTyper kit and in-house method, respectively (Table 3). In the Gram-positive bacteria group, correct identification rates were 100% (88/88) and 92% (81/88) for the SepsiTyper kit and in-house method, respectively. For Gram-negative bacteria, correct identification was achieved in 99% (78/79) and 95% (75/79) of the blood culture by the SepsiTyper kit and in-house method, respectively. Correct identification rates in the anaerobic bacteria group were 100% (12/12) and 75% (9/12) for the SepsiTyper kit and in-house method, respectively (Table 3).

**Table 3:** Correct identification rates by MS analysis using SepsiTyper kit and an in-house method

Microorganism group (N)	Correct identification rates (%)		
	SepsiTyper kit	In-house method	*p* Value
Gram negative bacteria (79)	99	95	< 0.0001
Gram positive bacteria (88)	100	92	< 0.0001
Yeasts (7)	86	43	0.24
Anaerobic bacteria (12)	100	75	< 0.005
Total (186)	99	90	< 0.0001

## Discussion

Rapid and accurate pathogen identification in blood cultures is very important for septic patients and has major consequences on sepsis morbidity and mortality rates. Currently, blood pathogens are cultured and then identified, thus the turnaround time for microorganism identification in positive blood cultures is about 24–48 h, a prolonged time during which the patient is treated with an empirical antibiotic regimen or is not treated at all. It was found that each hour of delay in appropriate antibiotic treatment over the first 6 h is linked to a 7.6% decrease in survival rate [6]. In patients with sepsis, empiric broad spectrum antimicrobial coverage is advocated. Rapid identification of blood pathogens enables adding appropriate therapy that was not included in the empiric regimen and implementation of one of the most important elements of antibiotic stewardship as well, more focused antibiotic treatment, which permits less promotion of antibiotic resistance [7]. Thus, reducing the time to pathogen recognition will remarkably improve patient outcomes and might assist in decreasing the use of broad-spectrum antibiotics.

Recently, a new technology, matrix-assisted laser desorption ionization-time of flight mass spectrometry (MALDI-TOF MS), enabled the identification of pathogens directly from blood cultures within a short time. This technology requires several preliminary steps for sample preparation and microorganism extraction from blood as purely as possible. For this purpose, several commercial kits and in-house methods have been developed. However, most of the in-house methods require preparation of lysis and washing buffers and multiple centrifugation steps. The commercial kits, which were developed in order to simplify preparation handling, are still multistep and expensive.

In the current study we described the evaluation of a rapid and easy-to-use method that allows pathogen identification from blood culture within 15 min. We compared our method to the SepsiTyper kit, which is recommended by the manufacturer of the Microflex LT MALDI-TOF MS system, and found high concordance (Pearson coefficient = 0.7, *p* <  0.0001).

A reliable identification is determined by a score ≥ 1.7 according to the manufacturer’s instructions. According to this cut-off, in the current study 88% (164/186) and 43.5% (81/186) of the isolates were reliably identified. However, if we do not stick to this cut-off and look at the final results, i.e., the name of identified organism in each method compared to the routine method, the correct identification rates were high, with 99 and 90% of the isolates correctly identified by the SepsiTyper kit and our in-house method, respectively.

Correlation between the methods was also high in sub-groups of identified bacteria, with Pearson coefficients of 0.77 (*p* <  0.0001), 0.67 (*p* <  0.0001), and 0.73 (*p* <  0.007) for Gram negative, Gram positive, and anaerobic bacteria, respectively. It was not surprising that no correlation was found for yeasts, due to their thick cell wall, making yeast identification by MS difficult. For more sensitive and accurate identification of yeasts, it is recommended to perform preliminary preparation steps in order to disturb the cell wall and liberate intracellular proteins.

Only 18 isolates out of 186 positive blood cultures were unidentified by our in-house method. Most of these isolates were Gram-positive bacteria, which are known to be difficult to identify by MS analysis [2, 8] and require pre-processing steps due to their thick cell wall.

Other unidentified isolates were *Candida albicans* and *Candida tropicalis*, which also require unique preparation. *Campylobacter fetus*, *Haemophilus influenzae*, and anaerobic bacteria were also not identified. The latter are all slow-growing bacteria, which may lead to low bacterial concentration. Additionally, we had a small sample size of the yeast and anaerobic bacteria subgroups. A future research should test whether addition of 1 μl of formic acid after deposit of microbial material on the MS target and before the addition of the matrix, as recommended by manufacturer for identification of Gram-positive bacteria and yeasts, will improve identification quality.

It is important to note that most of these unidentified isolates were identified using the SepsiTyper kit with relatively low scores.

Although MS analysis using the in-house method gave lower score results than using the SepsiTyper kit, most of the identification results were correct. Several studies have suggested lowering the cut-off score for successful identification below the manufacturer’s recommended cut-off (1.7) [8–13]. For example, Moussani et al. [9] suggested a cut-off of 1.4, when four successive proposals indicated different species belonging to the same genus.

In comparison with other laboratory-developed techniques, our in-house method has the advantage of being a quick and easy-to-perform procedure. While most of the in-house methods include buffer preparation and several centrifugation steps, our method requires only two centrifugation steps and the addition of saline only. In comparison with commercial kits, our in-house method is considerably time- and cost-saving. We should note that the small sample number and the use of only mono-microbial cultures limit our study results. However, it is known that MS analysis can be less accurate when the sample contains more than one bacteria/yeast species. Another limitation is the use of only one type of the available MS platforms.

## Conclusions

Our in-house method was found to be in good agreement with the SepsiTyper kit. In light of the fact that this method is very rapid and has significantly lower costs, we propose our in-house method for the direct identification of bacteria from blood cultures, especially in low-resource laboratories that are not equipped with the SepsiTyper kit. Additionally, it may be used as a first attempt to identify the microorganism. In cases of low identification quality such as in identification of Gram-positive bacteria or yeasts, we recommend to consider the addition of formic acid before matrix addition. This way, the use of the SepsiTyper kit can be limited to cases with unidentified microorganisms or with very low identification quality, therefore reducing time and costs of pathogen identification in blood cultures.

## Abbreviations

BC: Blood culture
HCCA: Alpha-cyano-4- hydroxycinnamic acid
HPLC: High Pressure/Performance Liquid Chromatography
Hrs: Hours
MALDI-TOF MS: Matrix-assisted laser desorption ionization–time of flight mass spectrometry
Min: minutes
ml: Milliliter
Rpm: Revolutions per minute
μl: Microliter

## References

[1] Bazzi AM, Rabaan AA, El Edaily Z, John S, Fawarah MM, Al-Tawfiq JA (2017). Comparison among four proposed direct blood culture microbial identification methods using MALDI-TOF MS. J Infect Public Health.

[2] Yonetani S, Ohnishi H, Ohkusu K, Matsumoto T, Watanabe T (2016). Direct identification of microorganisms from positive blood cultures by MALDI-TOF MS using an in-house saponin method. Int J Infect Dis.

[3] Seng P, Drancourt M, Gouriet F, La Scola B, Fournier P, Rolain JM (2009). Ongoing revolution in bacteriology: routine identification of Bacteria by matrix-assisted laser desorption ionization time-of-flight mass spectrometry. Clin Infect Dis.

[4] Singhal N, Kumar M, Kanaujia PK, Virdi JS (2015). MALDI-TOF mass spectrometry: an emerging technology for microbial identification and diagnosis. Front Microbiol.

[5] Morgenthaler NG, Kostrzewa M. Rapid identification of pathogens in positive blood culture of patients with sepsis: review and meta-analysis of the performance of the sepsityper kit. Int J Microbiol. 2015;2015:827416.10.1155/2015/827416PMC442677926000017

[6] Kumar A, Roberts D, Wood KE, Light B, Parrillo JE, Sharma S (2006). Duration of hypotension before initiation of effective antimicrobial therapy is the critical determinant of survival in human septic shock*. Crit Care Med.

[7] Barlam TF, Cosgrove SE, Abbo LM, MacDougall C, Schuetz AN, Septimus EJ (2016). Implementing an antibiotic stewardship program: guidelines by the Infectious Diseases Society of America and the Society for Healthcare Epidemiology of America. Clin Infect Dis.

[8] Barnini S, Ghelardi E, Brucculeri V, Morici P, Lupetti A (2015). Rapid and reliable identification of gram-negative bacteria and gram-positive cocci by deposition of bacteria harvested from blood cultures onto the MALDI-TOF plate. BMC Microbiol.

[9] Moussaoui W, Jaulhac B, Hoffmann A-M, Ludes B, Kostrzewa M, Riegel P (2010). Matrix-assisted laser desorption ionization time-of-flight mass spectrometry identifies 90% of bacteria directly from blood culture vials. Clin Microbiol Infect.

[10] Buchan BW, Riebe KM, Ledeboer NA (2012). Comparison of the MALDI Biotyper system using Sepsityper specimen processing to routine microbiological methods for identification of bacteria from positive blood culture bottles. J Clin Microbiol.

[11] Lagacé-Wiens PRS, Adam HJ, Karlowsky JA, Nichol KA, Pang PF, Guenther J (2012). Identification of blood culture isolates directly from positive blood cultures by use of matrix-assisted laser desorption ionization-time of flight mass spectrometry and a commercial extraction system: analysis of performance, cost, and turnaround time. J Clin Microbiol.

[12] Saffert RT, Cunningham SA, Mandrekar J, Patel R (2012). Comparison of three preparatory methods for detection of bacteremia by MALDI-TOF mass spectrometry. Diagn Microbiol Infect Dis.

[13] Barnini S, Brucculeri V, Morici P, Ghelardi E, Florio W, Lupetti A (2016). A new rapid method for direct antimicrobial susceptibility testing of bacteria from positive blood cultures. BMC Microbiol.

